This article has been retracted.

# CDX2/mir-145-5p/SENP1 Pathways Affect LNCaP Cells Invasion and Migration

**DOI:** 10.3389/fonc.2019.00477

**Published:** 2019-06-12

**Authors:** Jin-Hua He, Ze-Ping Han, Mao-Xian Zou, Meng-Ling He, Yu-Guang Li, Lei Zheng

**Affiliations:** ^1^Department of Laboratory Medicine, Central Hospital of Panyu District, Guangzhou, China; ^2^Department of Laboratory Medicine, Nanfang Hospital, Southern Medical University, Guangzhou, China

**Keywords:** miR-145-5p, CDX2, SENP1, prostate cancer, invasion, migration

## Abstract

**Background/Aims:** Recently, rapidly accumulating evidence has shown that microRNAs (miRNAs) are involved in human tumorigenesis, and the dysregulation of miRNAs has been observed in many cancers, including prostate cancer. miR-145-5p, an miRNA with reduced expression in prostate cancer cells, has been shown to have a tumor suppressive role in a variety of tumors. However, its underlying mechanism requires further elucidation.

**Methods:** A lentiviral expression vector for miR-145-5p was constructed and used to establish a stable cell line (LNCaP) expressing miR-145-5p. The cells were cultured normally and divided into the control group (control), negative control group (negative control), and test group (miR-145-5p). Inhibition of proliferation was measured by a WST-8 assay. The early apoptosis rate of cells was detected by flow cytometry. Clone formation ability was detected by a clone formation inhibition test. Cell invasion and migration capacity was detected by a Transwell assay. The relative expression levels of proteins were detected by western blotting. We constructed a nude mouse model of prostate cancer to observe the effect of miR-145-5p on the growth of transplanted tumors. TargetScan bioinformatics software was used to predict target genes regulated by miR-14-5p. ChIPBase was used to predict transcription factors with binding sites in the upstream promoter region of miR-145-5p. Quantitative reverse transcription PCR was used to detect the relative expression level of genes. A bifluorescence-reporter gene vector was constructed to confirm the regulation of target genes by miR-145-5p. We used 5′ rapid amplification of cDNA ends to confirm the transcription start site of miR-145-5p.Chromatin immunoprecipitation technology was used to detect the effect of transcription factors binding to miR-145-5p.

**Results:** The overexpression of miR-145-5p not only inhibited the proliferation, invasion, and migration of LNCaP cells but also promoted their early apoptosis. After overexpressing miR-145-5p, the expression of small ubiquitin-like modifier protein-specific protease 1 (SENP1), and caudal-related homeobox 2 (CDX2) protein was decreased in LNCaP cells. The transcription factor CDX2 bound to the miR-145-5p promoter region and inhibited its transcription. The transcription start site of miR-145-5p was located at a guanine residue 1,408 bp upstream of the stem-loop sequence. Upon overexpression, miR-145-5p could bind to the 3′-untranslated region of SENP1 to inhibit its translation.

**Conclusion:** These results suggested that CDX2 inhibits the expression of miR-145-5p, thereby relieving the inhibitory effect of miR-145-5p on the translation of SENP1 and affecting the invasion and migration of prostate cancer cells.

## Introduction

Prostate cancer has become the most common cancer for males in the United States. The mortality rate for prostate cancer is ranked second in the United States and third in Europe (1). In China, owing to the aging population, the incidence of prostate cancer continues to increase annually. Early diagnosis and treatment are correlated to the prognosis of prostate cancer. Therefore, study of the molecular mechanism of prostate cancer has become a recent focus of research.

MicroRNAs (miRNAs) have been shown to be closely related to the occurrence and development of prostate cancer (2). Previous studies have found that miR-145 and lncRNAPCGM1 could mutually regulate the proliferation of prostate cancer (3), and miR-145 was also shown to play a tumor suppressive role in neuroblastoma, osteosarcoma, uterine cancer, and prostate cancer (4). However, the underlying molecular mechanism needs to be explored further. The expression of small ubiquitin-like modifier (SUMO)-specific protease 1 (SENP1) was previously shown to be up-regulated in prostate cancer cells. By utilizing the bioinformatics software TargetScan, we found that SENP1 was one of the target genes regulated by miR-145-5p. We also found that most of the core promoter regions of miRNA genes contained a TATA box and cell-specific transcriptional regulatory elements that could affect miRNA expression (5). ChIPBase software predicted that the transcription factor (TF) caudal-related homeobox 2 (CDX2) could bind to miR-145-5p at several binding sites in its upstream promoter region. Therefore, in this study, we established a stable LNCaP cell line overexpressing miR-145-5p in order to observe the effect of miR-145-5p on cell proliferation, invasion, and migration, and further clarify the underlying molecular mechanism.

## Methods

### Cell Culture

293T cells, non-cancerous RWPE-1 (human prostate epithelial cell line) cells, and cancerous LNCaP (androgen-sensitive human prostate adenocarcinoma cells) cells were purchased from the Shanghai Institute of Cell Biology (Shanghai, China). The cell lines were cultured in Dulbecco's modified Eagle's medium (DMEM; Gibco BRL, Grand Island, NY) containing 10% fetal bovine serum (FBS, HyClone; Invitrogen, Camarillo, CA), 100 U/mL penicillin (Invitrogen), and 100 μg/mL streptomycin (Invitrogen). The cells were maintained in a humidified incubator at 37°C with 5% CO_2_. All cell lines were passaged for < 6 months (3).

### Vector Construction, Virus Packaging, and Preparation of Stable miR-145-5p Cell Lines

Human cDNA was used as the template. The upstream and downstream primers were designed to contain the following cleavage sites: Hsa-miR-145-5p *Eco*RI F: 5′-ccggaattcCGCCAGAGGGTTTCCGGTACTTTTC-3′; and Hsa-miR-145-5p *Bam*HI R: 5′-cgcggatccCATCCAGCCTCACAGGGATGTTA-3′. The PCR products were sequenced. After double digestion of the PCR products and lentiviral vector, the lentiviral vector was purchased from Jima Biotech Co., Ltd (Shanghai, China). They were ligated overnight. The lentiviral vector and packaging plasmid were mixed in a certain proportion and transfected into 293T cells. At 6 h of transfection, the medium was changed. Virus-containing medium was collected after 48 h, concentrated, and viral titer was measured. LNCaP cells were then infected with the virus in the presence of Polybrene to enhance the rate of infection. Empty vector-infected LNCaP cells were used as the negative control (NC) group. At 48 h after infection, puromycin was added for the selection of successfully transfected LNCaP cells (6). A quantitative reverse transcription PCR (qRT-PCR) assay was used to detect the relative expression of miR-145-5p (6).

### Cell Transfection

LNCaP cells were seeded at a density of 2.0 × 10^5^ cells/well in a 6- or 96-well culture plate (COSTAR#3516; Corning, Inc., Corning, NY) and transfected when cell confluency reached 70%. RNA Lipofectamine 2000 (Invitrogen) was used to transfect the cells with small interfering RNAs (siRNAs) to SENP1 or CDX2 according to the manufacturer's instructions. Discarded the transfection after 6 h.Then, the cells were washed with serum-free DMEM, and cultured in DMEM supplemented with 10% FBS. At 48 h after transfection, the cells were harvested for further studies. The siRNAs were designed and synthesized by Shanghai GenePharma Co., Ltd. (Shanghai, China). SiRNA for SENP1 sense: 5′-GAAACAGCCGAAGCCUUUAdTdT-3′; anti-sense: 5′-UAAAGACUUCGGCUGUUUCdTdT-3′; and siRNA for CDX2: sense 5′-GAAGAAGTTGCAGCAGCAA-3′; anti-sense: 5′-UUGCUGCUGCAACUUCUUC-3′.

### Cell Proliferation Assay

The proliferation of LNCaP cells was evaluated by a Cell Counting Kit-8 assay (CCK-8; Dojindo, Kumamoto, Japan) according to the manufacturer's instructions. The cells were seeded into 96-well plates at 5.0 × 10^4^ cells/mL and divided into the following groups: LNCaP-miR-145-5p (stably transfected miR-145-5p), LNCaP-NC (empty virus infection), and LNCaP (not infected with the virus), and serum-free DMEM medium was added for 6 h. The cells were cultured for 1, 2, and 3 days before the addition of 10 μL CCK-8 (5 mg/mL) to the culture medium in each well. After incubation for 2 h at 37°C, absorbance at 450 nm was measured using a multifunctional microplate reader (excitation wavelength at 450 nm, reference wavelength at 655 nm; Bio-Rad, Hercules, CA, USA), and the inhibition of cell proliferation was calculated (6).

### Flow Cytometry Assay

LNCaP cells were seeded at 1.0 × 10^6^/ml in 24-well plates (Costar, Corning, Inc.) in serum-free DMEM for 48 h. Then, 500 μL of the appropriate growth medium containing 20% FBS was added to each well. The cells were harvested, washed twice with phosphate-buffered saline (PBS), fixed with 70% ethanol, and treated with RNase A (1 mg/mL). Finally, the cells were double-stained with a fluorescein isothiocyanate-conjugated annexin V and propidium iodide (PI) solution (50 μg/mL). For each sample, data from ~10,000 cells were recorded in the list mode on logarithmic scales. Apoptosis and necrosis were analyzed by quadrant statistics on double negative, annexin V-positive/PI-negative, annexin V-negative/PI-positive, and double-positive cells (6).

### Colony Formation Assay

The cells were seeded at a density of 100 cells/well in a 6-well plate (6 cm, Costar; Corning, Inc.). The cells were grouped as described above and incubated at 37°C for 12–14 days. The cells were fixed for 15 min in 3:1 (v/v) methanol-to-acetic acid and stained for 15 min with 0.5% (w/v) crystal violet (Sigma-Aldrich, St. Louis, MO) in methanol. After staining, colonies containing more than 10 cells were observed under a microscope. These experiments were performed in triplicate.

### Transwell Assay

Matrigel was diluted in a pre-cooled serum-free medium at a volume ratio of 1:3; 40 μL was added into a precooled Transwell chamber and incubated at 37°C for 2 h. Then, the excess liquid was removed from the chamber, 100 and 600 μL serum-free medium was added to the upper and lower chamber, respectively, and incubated overnight at 37°C. The next day, the cells were transfected, and 1.0 × 10^5^ cells were counted. Then, the cells were resuspended in 100 μL serum-free DMEM-F12 medium and added to the upper Transwell chamber, and 600 μL complete medium was added to the lower chamber. After incubation at 37°C in 5% CO_2_ for 24 and 48 h, the chamber was removed, the cells were wiped with a cotton swab, and the cells were observed and photographed under an inverted microscope.

### *In vivo* Treatment

A total of 18 androgen BALB/c nude mice (weight, 18–20 g) were purchased from the Guangdong Experimental Animal Center (animal production license no: 44007200008792). Three cell lines (LNCaP-miR-145, LNCaP-NC, and LNCaP) were digested with 0.25% trypsin, washed with PBS, counted by trypan blue staining, and adjusted to a concentration of 1.0 × 10^7^ cells/mL, and 0.1 mL aliquots were used each time. After mixing with Matrigel matrix (Beijing Xia Si Biotechnology Co., Ltd., Beijing, China), the cells were injected subcutaneously between the abdominal ribs of specific pathogen free-grade male nude mice aged 4–6 weeks. The tumor growth rate of the tumor-bearing mice was observed daily (volume and weight) when tumor growth became visible, and a tumor growth curve was plotted (6).

### Western Blot Analysis

Human LNCaP cells were seeded in 12-well plates at a density of 1.0 × 10^6^ cells/well in a total volume of 1 mL. After 48 h, each group of cells was lysed, and according to the cell lysis buffer (RIPA) instructions, cellular protein was extracted. Protein quantification was performed using a BCA Protein Quantification Kit, and each sample was adjusted to the same concentration. Then, the samples were added to the loading solution and boiled for 5 min. Discontinuous polyacrylamide gel electrophoresis (10% polyacrylamide gel and 5% polyacrylamide concentrate) was conducted at a voltage 80 V, and this was changed to 120 V for 40 min after the samples entered the separation gel. Then, the protein bands on the gel were transferred to a nitrocellulose membrane and semi-dry transfer film at 15 V for 18 min. Afterwards, the membrane was washed with tris-buffered saline with Tween 20 (TBST) for 5 min, blocked in 5% bovine serum albumin blocking buffer at room temperature for 1 h, and washed 3 times with TBST for 5 min. The membrane was incubated with a primary antibody overnight at 4°C, and the membrane was washed three times with TBST for 5 min. The membrane was incubated with a secondary antibody for 1 h at 37°C, and the membrane was washed three times with TBST for 5 min. An electrochemiluminescence reagent was added and developed. BI-2000 image analysis software was used to analyze the integral optical density, with glyceraldehyde 3-phosphate dehydrogenase as the internal reference (6).

### Luciferase Reporter Assay

The full sequence or 3′-untranslated region (3′UTR) of the gene was obtained by PCR amplification and cloned separately into the multiple cloning site of the psi-CHECK^TM−2^ luciferase miRNA expression reporter vector. 293T cells were transfected with an miRNA mimic, miRNA inhibitor, control miRNA, control miRNA inhibitor, or empty plasmid (50 nM; RiboBio, Guangzhou, China) using Lipofectamine 2000 according to the manufacturer's instructions. Nucleotide-substitution mutation analysis was carried out using direct oligomer synthesis of the full sequences or 3′UTR. All constructs were verified by sequencing. Luciferase activity was measured using a Dual Luciferase Reporter Assay System Kit (Promega, Madison, WI) on a Tecan M200 luminescence reader according to the manufacturer's instructions (7).

### Chromatin Immunoprecipitation (ChIP) Assay

LNCaP cells were treated with formaldehyde and incubated for 10 min to generate DNA-protein cross-links. Then, cell lysates were sonicated to generate chromatin fragments of 200–300 bp, and immunoprecipitated with CDX2 or IgG as control. The precipitated chromatin DNA was recovered and analyzed by qRT-PCR. Gene-specific primers were designed according to the sequence of CDX2 (5′-CGGACACTTGCCATTAATACT-3′ and 5′-GGCAACTTCCTCTCTGATAAC-3′). qRT-PCR was performed to measure target DNA levels in the purified DNA products (6).

### 5′ Rapid Amplification of cDNA Ends (5′RACE)

LNCaP cell RNA was extracted and dephosphorylated, and tobacco acid pyrophosphatase was used to remove the 5′ cap structure of the mRNA, which retained a phosphate group, at 37°C for 1 h. The product was reacted with the 5′RACE adaptor at 65°C for 5 min, and reverse transcription of the cDNA was conducted using reverse transcriptase. In the first outer primer PCR, PCR was carried out with the inner primer, and the PCR product was ligated with a T vector. PCR was performed using an inner primer (5′-GGGATTCCTGGGAAAACTGGACC-3′) and outer primer (5′-GACCTCAAGAACAGTATTTCCAGG-3′) that were specific for the miR-145-5p coding sequence. Then, the PCR product was cloned and sequenced, the sequencing results were compared with the genomic sequences, and the gene transcription initiation site was determined.

### Data Analysis

All results are the average of at least three independent experiments from separately treated and transfected cultures. Data are expressed as the mean ± standard deviation. Statistical comparisons were performed using one-way analysis of variance and a *t*-test. A *P* < 0.05 was considered statistically significant.

## Results

### Construction of an LNCaP Cell Line Overexpressing miR-145-5p

The pre-sequence of miR-145-5p was cloned into the pLVX-mCMV-ZsGreen-puro vector, and 293T cells were co-transfected with the envelope plasmid pHelper 1.0 and the packaging plasmid pHelper 2.0. Then, the virus titer was measured at 1.25 × 10^8^ TU/mL using a dilution method. At MOI = 50, the rlv-miR-145-5p virus was added to LNCaP cells (Figures 1A,B). Fluorescence microscopy was used to confirm that the constructed LNCaP cells overexpressed miR-145-5p (Figures 1C,D). qRT-PCR was used to detect the relative expression of miR-145-5p (Figure 1E). The results showed that the relative expression of miR-145-5p was higher in the miR-145-5p-infected cells than in the NC group, indicating the successful construction of LNCaP cell lines overexpressing miR-145-5p and laying the foundation for the study of its function.

**Figure 1:** Establishment of a miR-145-5p-overexpressing LNCaP cell line. **(A)** PCR amplification of miR-145-5p. M1: 1 kb DNA marker; 1: negative PCR amplification; 2: miR-145-5p PCR amplification product (466 bp); 3: negative PCR amplification; M2: DL2000 DNA marker. **(B)** The miR-145-5p PCR product was ligated into the lentiviral vector and identified by double digestion. M1: 10 kb DNA marker; 1: undigested plasmids; 2: Plasmids were digested by double enzymes; M2: DL 2000 DNA marker. **(C)** 293T cell line stably transfected with the virus. **(D)** LNCaP cell line stably transfected with negative control for miR-145-5p (7). **(E)** Detection of the relative expression of miR-145-5p by qRT-PCR; ^Δ^*P* < 0.05 vs. the control and NC groups.

### Overexpression of miR-145-5p Inhibits LNCaP Cell Proliferation and Promotes Early Apoptosis

The effect of miR-145-5p expression on LNCaP cell proliferation was investigated. a CCK-8 assay revealed that the inhibitory rate of proliferation was significantly increased in a time-dependent manner. The inhibitory rate of proliferation was significantly higher in the treatment group than in the NC group (*P* < 0.05, Figure 2A). Flow cytometry was used to detect the early apoptosis rate after 48 h. It was found that the early apoptosis rate was significantly increased in LNCaP cells overexpressing miR-145-5p compared with the NC and control groups (*P* < 0.05, Figures 2B,C). A clone formation assay revealed that the clonogenic ability of LNCaP cells overexpressing miR-145-5p was significantly decreased (*P* < 0.05, Figures 2D,E). Furthermore, the three cell lines (LNCaP-miR-145-5p, LNCaP-NC, and LNCaP) were injected subcutaneously between the nude mice, and the resultant tumor volumes were observed. It was found that tumor growth was slow and tumor volume was significantly reduced in the LNCaP-miR-145-5p group compared with the LNCaP-NC and LNCaP groups (*P* < 0.01, Figures 2F–H). These results indicated that miR-145-5p overexpression could inhibit the proliferation of LNCaP cells and promote the early apoptosis rate.

**Figure 2:** Effects of miR-145-5p overexpression on the proliferation and apoptosis of LNCaP cells. **(A)** The inhibitory rate of proliferation was detected by a CCK-8 assay; ^*^P < 0.05, ^**^P < 0.05, ^***^P < 0.01 compared with the NC group. **(B)** Cells undergoing early apoptosis were detected by annexin V/PI double staining. **(C)** Early cell apoptosis rate; ^*^P < 0.05, ^**^P < 0.05 compared with the NC and control groups. **(D)** Cell clonogenic ability was evaluated by a clone formation assay. **(E)** Cell clone formation rate; ^*^P < 0.05, ^**^P < 0.05 compared with the NC and control groups. **(F)** Tumor formation in nude mice. **(G)** Photographs of tumors from each group. **(H)** Tumor volume growth curve of each group of nude mice; ^*^P < 0.01, ^**^P < 0.05 compared with the NC and control groups.

### Overexpression of miR-145-5p Inhibits LNCaP Cell Invasion and Migration

The effect of miR-145-5p overexpression on the invasion and migration of LNCaP cells was investigated. At 48 h after the successful transfection of LNCaP cells with miR-145-5p, LNCaP cell invasion and migration were decreased, and the number of cells that invaded and migrated was significantly different in the miR-145-5p group compared with the NC group (*P* < 0.05, Figures 3A–D). The expression levels of invasion- and migration-related proteins were detected by western blotting (8–12). These results revealed that E-cadherin protein expression was increased, while the expression of β-catenin, MMP2, and MMP9 was decreased. The difference in the expression levels of E-cadherin, β-catenin, MMP2, and MMP9 was not significantly different between the blank control group and NC group (Figure 3E). The results showed that miR-145-5p overexpression could inhibit the invasion and migration of LNCaP cells.

**Figure 3:** Effect of miR-145-5p overexpression on cell migration and invasion. **(A)** A cell migration assay was performed on LNCaP cells overexpressing miR-145-5p. **(B)** A cell invasion assay was performed on LNCaP cells overexpressing miR-145-5p. **(C)** The number of migrated cells in the control, NC, and miR-145-5p groups; ^*^P < 0.05 compared with the NC and control groups. **(D)** The number of invaded cells in the control group; ^*^P < 0.05 compared with the NC and control groups. **(E)** The expression of E-cadherin, β-catenin, MMP2, and MMP9 protein detected by western blotting.

### Binding of miR-145-5p to the 3′UTR of SENP1

TargetScan (Human 6.2 version), an miRNA target gene prediction software, predicted the presence of a miR-145-5p binding site on SENP1 at 516–522 bp of the 3′UTR (Figure 4A). SENP1 is a member of the SUMO protease family and has an important role in the regulation of androgen receptor-dependent transcription and hypoxia signaling (13). SENP1 might be a prognostic marker and therapeutic target for metastasis in prostate cancer, and might contribute to malignant progression in LNCaP (14). In order to determine whether these previously observed effects were regulated via the 3′UTR of SENP1, a luciferase reporter plasmid containing the 3′UTR of SENP1 was constructed. LNCaP cells were co-transfected with miR-145-5p mimics and psi-CHECK^TM−2^-SENP1-3′UTR to detect the miR-145-5p binding site in the 3′UTR of SENP1. Co-transfection of LNCaP cells with miR-145-5p mimics and psi-CHECK^TM−2^-SENP1-3′UTR significantly inhibited luciferase activity (*P* < 0.05, Figure 4B). However, co-transfection of LNCaP cells with miR-145-5p mimics and psi-CHECK^TM−2^-mutated (mut)-SENP1-3′UTR had little effect on luciferase activity (*P* > 0.05, Figure 4C). The above results demonstrated that miR-145-5p exerted a regulatory effect by binding to the 3′UTR of SENP1.

**Figure 4:** miR-145-5p binds directly to the 3′UTR of SENP1. **(A)** The target sequences for miR-145-5p within the 3′UTR of SENP1. **(B)** Comparison of luciferase activity in cells of different groups that were co-transfected with the 3′UTR of SENP1. ^*^P < 0.05. **(C)** Luciferase activity in cells of different groups that were co-transfected with mut-3′UTR of SENP1. ^*^P > 0.05.

### Transcription Initiation Site for miR-145-5p Determined by 5′RACE Assay

Specific primers for the miR-145-5p gene were designed for PCR amplification. An amplification product of 1,400 bp was obtained and cloned into the T vector, followed by enzyme digestion. The final sequencing result indicated that the transcription initiation site of miR-145-5p was located at 1,408 bp upstream of the stem-loop sequence (Figure 5).

**Figure 5:** Transcription initiation site for miR-145-5p determined by 5′RACE assay. **(A)** DNA electrophoresis of 5′RACE products. M1: DL2000 DNA marker; 1: amplified with outer primer bands; 2: amplified with inner primer bands; M2: 10 kb DNA marker. **(B)** DNA electrophoresis of the amplified miR-145-5p products constructed into the T vector before and after double digestion. M1: DL2000 DNA marker; 1: empty vector; 2: identification of recombinant plasmids by double enzyme cleavage gel; M2: 10 kb DNA marker. **(C)** The structure of the miR-145-5p promoter region with the possible binding site for CDX2.

### Binding of CDX2 to the Promoter Region of miR-145-5p

For CDX2, an intestine-specific TF with a role in the proliferation of porcine intestinal epithelial cell line one, novel intestinal nutrient transporter genes activated by CDX2 were screened (15). The transcription initiation site of miR-145-5p has been predicted use jaspar software (http://jaspar.genereg.net/). In order to confirm further whether CDX2 could bind to the promoter region of miR-145-5p, a ChIP assay was performed to verify the predicted binding site for CDX2 on miR-145-5p, which was located at 383 bp upstream of the transcription initiation site of miR-145-5p. DNA electrophoresis suggested that CDX2 protein was detected in a product from the ChIP assay, but not in the NC group. qRT-PCR revealed that the relative gene expression of CDX2 amplified by the CDX2 ChIP F/R primer was ~17-fold higher than in the negative group, suggesting that the DNA isolated using the anti-CDX2 antibody contained the predicted miR-145-5p promoter sequence. These results indicated that CDX2 could bind directly to the promoter sequence of miR-145-5p (Figure 6).

**Figure 6:** ChIP assay to assess CDX2 binding to the promoter region of miR-145-5p. **(A)** DNA electrophoresis of sonicated LNCaP cells. M: DL2000 DNA marker; 1, DNA extracted from LNCaP cells. **(B)** DNA electrophoresis of the products from the ChIP assay. M: DL2000 DNA marker; 1, LNCaP-input-ChIP-CDX2 (167 bp); 2, LNCaP-(-)-ChIP-CDX2; 3, LNCaP-(+)-ChIP-CDX2 (167 bp); M: DL2000 DNA marker. **(C)** miR-145-5p promoter DNA sequence detected by qRT-PCR was immunoprecipitated using an anti-CDX2 antibody; ^*^P < 0.05 compared with the IgG group.

### CDX2 Inhibits the Expression of miR-145-5p, Which Negatively Regulates the Expression of SENP1

In order to further investigate the relationship among CDX2, miR-145-5p, and SENP1, the expression of miR-145-5p and SENP1 was compared in prostate cancer cells and normal prostate epithelial cells. The results showed that CDX2 and SENP1 were highly expressed in prostate cancer epithelial cells, while miR-145-5p expression was decreased. miR-145-5p overexpression down-regulated the expression of CDX2 and SENP1 in prostate cancer cells. At 48 h after transfection of LNCaP cells with siRNA-SENP1, miR-145-5p, and CDX2 expression was increased. When CDX2 expression was reduced in LNCaP cells, miR-145-5p expression increased, and the expression of SENP1 decreased. These results showed that CDX2 could inhibit miR-145-5p expression, which negatively regulated the expression of SENP1 (Figure 7).

**Figure 7:** CDX2 inhibits miR-145-5p expression, which negatively regulates the expression of SENP1. **(A)** SENP1 expression levels in different treatment groups. **(B)** CDX2 expression levels in different treatment groups. **(C)** miR-145-5p expression levels in different treatment groups. **(D)** CDX2 and SENP1 protein expression in different treatment groups detected by western blotting.

## Discussion

In this study, we constructed a miR-145-5p lentiviral expression vector, and established a stable LNCaP cell line overexpressing miR-145-5p. miR-145-5p overexpression inhibited the proliferation, invasion, and migration of LNCaP cells *in vitro* and *in vivo*. These results suggested that miR-145-5p might play an important role in the growth and metastasis of prostate cancer. Our findings are consistent with the report by Avgeris et al. (16). In order to study its molecular mechanism, a dual-luciferase reporter gene vector was constructed. miR-145-5p could bind to the 3′UTR of SENP1, and negatively regulated its expression. The results are consistent with the findings of Wang et al. (17). It was also reported that miR-145-5p could suppress cell proliferation, invasion, and migration, and induce the apoptosis of CHL-1 and VMM917 melanoma cells by inhibiting the MAPK and PI3K/AKT pathways (18). miR-145-5p might also function as a cardiac-protective molecule in myocardial ischemic injury by ameliorating inflammation and apoptosis via the negative regulation of CD40 (19). miR-145 has been shown to mediate epithelial-mesenchymal transition by targeting Snail, suggesting that it might be a novel epithelial-mesenchymal transition-regulating TF involved in the progression of osteosarcoma (20). miR-145 can also negatively regulate the invasion of cancer cells through targeting N-cadherin by binding directly to its 3′UTR. The silencing of N-cadherin further inhibited the invasion and migration of LAC cells, which was similar to the effect of overexpressing miR-145 (21). miR-145 was also shown to be capable of inducing cervical tumorsphere differentiation by enzymolyzing TFs, which makes it a potential therapeutic target for cervical carcinoma. miR-145 promotes hepatic stem cell activation and liver fibrosis by targeting KLF4 (22). These results together suggest that miR-145-5p may play an important tumor suppressive role in a variety of tumors, which indicates a possible future direction for the development of clinical targeted gene therapy for cancer.

MicroRNAs are small molecular RNAs that regulate gene expression at the post-transcriptional level, which can comprise TFs, in which their interaction with the target gene is adjusted, constituting a gene expression regulation network (23). In the miRNA-TF common target gene regulation process, TFs can regulate miRNAs, which in turn can be regulated by miRNAs, forming a feed-forward loop (24). In the present study, we found that the transcription initiation site of miR-145-5p was located at 1,408 bp upstream of the stem-loop sequence, and the TF CDX2 bound to the promoter region and inhibited miR-145-5p transcription (Figure 5). miRNAs and TFs have a fine regulatory effect on the expression of target genes in intact gene transcription-transcriptional regulatory networks (25). For example, Bcl6 can regulate miR-21 expression by binding to Stat3-binding elements on miR-21 to down-regulate miR-21 expression, promote Th2 differentiation through T-cell pathways, and inhibit the Th2-type inflammatory response (26). The TF SNAI2 represses the expression of miR-203 to promote epithelial-mesenchymal transition and tumor metastasis (27). Another study revealed that miR-202 is activated by E2F1, which in turn down-regulates MYCN protein expression in the neuroblastoma LAN-5 cell line (28). Thus, TFs interact with miRNAs to form a feed-back loop to regulate gene expression.

## Conclusion

In conclusion, our results demonstrated that the TF CDX2 could bind to the miR-145-5p promoter region to inhibit its transcription. The transcription start site of miR-145-5p was located at a guanine residue 1,408 bp upstream of the stem-loop sequence. After overexpressing miR-145-5p, miR-145-5p could bind to the 3′UTR of SENP1 to inhibit SENP1 protein translation. In summary, CDX2 inhibited miR-145-5p expression, thereby relieving the inhibitory effect of miR-145-5p on the translation of SENP1 and affecting the invasion and migration of prostate cancer cells (Figure 8). This provides a potential clue to the pathogenesis of prostate cancer and suggests a possible future direction for the development of clinical targeted gene therapy for cancer.

**Figure 8:** Molecular mechanism of the CDX2/miR-145-5p/SENP1 regulatory axis affecting the invasion and migration of prostate cancer cells.

## Ethics Statement

This study was carried out in accordance with the recommendations of the Medical Animal Care and Welfare Committee of Southern Medical University. The protocol was approved by the Medical Animal Care and Welfare Committee of Southern Medical University.

## Author Contributions

J-HH performed the experiments and analyzed the data. Z-PH wrote the manuscript. Y-GL designed the study and revised the manuscript. M-XZ provided the reagents. M-LH performed the experiment. All authors read and approved the final manuscript.

### Conflict of Interest Statement

The authors declare that the research was conducted in the absence of any commercial or financial relationships that could be construed as a potential conflict of interest.

## Abbreviations

miR: microRNA
CCK-8: Cell Counting Kit-8
TF: transcription factor
qRT-PCR: quantitative reverse transcription polymerase chain reaction
3′UTR: 3′-untranslated region
ChIP: chromatin immunoprecipitation
SUMO: small ubiquitin-like modifier
SENP1: protein-specific protease 1
CDX2: caudal-related homeobox 2
DMEM: Dulbecco's modified Eagle's medium
FBS: fetal bovine serum
NC: negative control
siRNA: small interfering RNA
PBS: phosphate-buffered saline
PI: propidium iodide.
